The article "Managing the Gate Assignment Problem in the Hub Airport with Satellite Halls: A Transfer Demand-Oriented Approach" was retracted in 2023. Reasons: unreliable results or conclusions; concerns about the data; concerns about the peer review; concerns about the citations.

# Managing the Gate Assignment Problem in the Hub Airport with Satellite Halls: A Transfer Demand-Oriented Approach

**DOI:** 10.1155/2022/5087941

**Published:** 2022-04-25

**Authors:** Runfa Wu, Wenliang Zhou, Linhuan Zhong, Yihan Liu

**Affiliations:** School of Traffic and Transportation Engineering, Central South University, Changsha, Hunan 410075, China

## Abstract

This study focuses on managing the gate assignment in the hub airport with both main terminal and satellite halls. We first formulate the gate assignment problem (GAP) as a binary linear programming model with multi-objective functions, where the practical constraints, e.g., gate time conflict and gate compatibility, are considered. Then, we incorporate the impact of gate assignment on transfer passengers and formulate the transfer demand-oriented gate assignment problem (TGAP) as a nonlinear model. A linearization approach and a heuristic approach are designed to solve the TGAP model. A case study is conducted based on the practical data of the Shanghai Pudong International Airport, where a comparison between the results of GAP and TGAP by the two proposed approaches is demonstrated. It shows that the proposed TGAP model and solution approaches can not only enhance the service for transfer passengers but also improve the gate utilization efficiency in the hub airport.

## 1. Introduction

Global air passenger demand and airport construction have experienced rapid growth over the past few decades, and passenger demand still grew steady in 2019 before the COVID-19 pandemic [1]. Driven by the recovery in domestic markets in China, many hub airports have returned to pre-pandemic levels in passenger demand and flight numbers; e.g., Shanghai Pudong International Airport was handling 110,000 domestic travelers and 900 domestic flights every day in March 2021, which are both more than that of 2019 [2]. As the import part of the hub-and-spoke system in air transportation, hub airports are experiencing rapid growth in passenger demand and flight numbers. To release operating pressure and provide better airplane/flight service and passenger service, many hub airports have built satellite halls connected with terminals by underground walkways or mass rapid transit (MRT) systems. This raises new challenges for efficient operations and passenger services in the hub airport.

Gates are a scarce resource at hub airports, facing intense air traffic and passenger demand pressure [3]. The gate operation connects air traffic (timetable and airplane service), passenger service, and ground operations (including crew assignment), which makes it critical for efficient airport operations. The gate assignment problem (GAP) is to assign airplanes/flights to suitable boarding gates or the apron at the airport on an operating period (usually one day), according to the given flight timetable and airplane fleet assignment, also taking into account the airport layout, gate compatibility, airplane types, and so on. The typical objectives of GAP usually include two aspects, minimizing the operating costs and maximizing the efficiency of gate resources for airport operators; and maximizing satisfaction for passengers. The GAP has been extensively studied as one of the most important problems in the daily operations of the airport, and see [4, 5] for a detailed literature review, and we give an overview from airport and passenger perspectives.

The article "Managing the Gate Assignment Problem in the Hub Airport with Satellite Halls: A Transfer Demand-Oriented Approach" was retracted in 2023. Reasons: unreliable results or conclusions; concerns about the data; concerns about the peer review; concerns about the citations.

From the airport operator perspective, the main objectives for GAP are efficient utilization of gate resources and reducing operating costs. Since the parking positions in the apron are usually far from the terminals and passengers need to take the shuttle bus. If airplanes are assigned to the apron, it will increase the waiting time of passengers and operation costs due to potential effects on ground operations and crew assignment. The most common objective in GAP literature is to minimize the airplanes/flights assigned to the apron (Ding et al. [6], Dorndorf et al. [7, 8], Drexl and Nikulin [9], Deng et al. [10]). Some studies aim to minimize the total delay of airplanes when the airport is busy (Lim et al. [11], Kaliszewski et al. [12]). Moreover, as Karsu et al. [13] point out, hub airports may need to handle different types of flights (domestic/international) and airplanes, so minimizing the moves/costs of towing when airplanes need to move from a gate to another is also considered in the literature (Benlic et al. [14], Kumar and Bierlaire [15], Yu et al. [16]). We consider the gate compatibility instead of the towing operation in this study to capture the matching between airplane/flight types and gate facilities. It was also modeled in the objective function of Benlic et al. [14] and Neuman and Atkin [17]. Following the conclusion that the airport controls gate use will ensure they are used most efficiently in the survey of Gillen and Lall [18], we also consider the integrated operating of gates in terminal and satellite halls in the hub airport and include minimizing the number of used gates in the objective function.

Gate assignment also affects the passenger service quality in the airport [11], and it may influence the walking distance, waiting time, and transfer service of passengers. The consideration of passengers in the literature is mainly reflected in the objective function. Hub airports in metropolitan usually have multiterminals, and it may take a lot of time/distance to get the specific gate or transfer between gates, and many studies contribute to GAP to minimize walking time/distance of passengers. Bohr [19] proposed binary linear programming to minimize the passenger walking distance and solved it by the primal-dual simplex algorithm. Karsu et al. [13] formulated a mixed-integer nonlinear programming model for GAP to minimize the total walking distance of all passengers and the number of airplanes assigned to the apron and then proposed exact and heuristic approaches to solve it. Interested readers can also refer to Drexl and Nikulin [9], Haghani and Chen [20], Dell'Orco et al. [21], and Mokhtarimousavi et al. [22]. Besides, Yan and Huo [23] and Yan and Tang [24] are focused on minimizing the total passenger waiting time in GAP. However, from the survey of Entwistle [25], over 60% of passengers plan to shop in the airport, which means minimizing the waiting time is not always the objective of passengers, at least for some of them. Daş [26] proposed a multi-objective model to increase the shopping revenues in the airport through gate assignment, by minimizing the total passenger walking distance and assigning passengers to gates near the shop. We consider the transfer time budget of passengers in this study and propose a more comprehensive way to measure service for transfer passengers. A comparison with some abovementioned major-related studies is shown in Table 1.

The article "Managing the Gate Assignment Problem in the Hub Airport with Satellite Halls: A Transfer Demand-Oriented Approach" was retracted in 2023. Reasons: unreliable results or conclusions; concerns about the data; concerns about the peer review; concerns about the citations.

In this study, we focus on the impacts of gate assignment on the service of transfer passengers in the hub airport with satellite halls. We proposed a novel transfer demand-oriented objective function considering the transfer time budget, together with objective functions of the airport operator, to explore the trade-off between airport operations and passenger service. Besides, we propose two optimization models, namely a binary linear programming model for gate assignment problem (GAP) and a nonlinear model for transfer demand-oriented gate assignment problem (TGAP). A linearization approach and a heuristic approach are designed to solve the TGAP model, and then, case studies are performed using the data of Shanghai Pudong International Airport.

The remainder of this study is organized as follows. In Section 2, we give a detailed description of GAP and TGAP. The corresponding mathematic models are formulated in Section 3. Then, Section 4 develops the linearization approach and heuristic approach to solve the model. Case studies are illustrated in Section 5, and Section 6 concludes the study.

## 2. Problem Statement and Assumptions

### 2.1. Problem Statement

We consider a hub airport with the main terminal and several satellite halls, illustrated in Figure 1. Gates are available in both the terminal and satellite halls and integrated assigned by the airport operator, denoted by *g* ∈ *G*. Passengers can travel between the terminal and satellite halls via the MRT system. As shown in Figure 1, the airport also has parking positions for airplanes at the apron, denoted by *G*′, in case an airplane could not be assigned to a gate in the terminal or satellite halls.

The article "Managing the Gate Assignment Problem in the Hub Airport with Satellite Halls: A Transfer Demand-Oriented Approach" was retracted in 2023. Reasons: unreliable results or conclusions; concerns about the data; concerns about the peer review; concerns about the citations.

The research period in this study is denoted by [*T*_1_,  *T*_2_]  (i.e., one day or one week) and discretized into equal-length time intervals *t*, and let *t* ∈ *T*. Some airplanes land and take off at the airport in this period, they occupy the gates for passenger arrivals and departures, and the set of airplanes is denoted by *I*. The services that provided by airplanes to transport passengers between airports are called a *flight*. For a specific airport, one airplane serves two flights, and we assume that the related flights of each airplane and the timetable are given. In Figure 2, we show the relationship between airplanes and related flights it serves. An airplane *i* ∈ *I* is considered, and it serves two flights: one arriving flight with arrival time *a*_*i*_ and one departing flight with departure time *d*_*i*_, and it needs to occupy a gate *g* ∈ *G* or a parking position *g* ∈ *G*′ during the time period [*a*_*i*_, *d*_*i*_]. Besides, the type of airplanes (wide/narrow-body) and related flights (domestic/international) are also given. Since the correspondence between aircrafts and flights is given, it is possible to model by either airplane or flight, and we use the airplane for modeling in this study.

As for the utilization of gates, the first thing to consider is time conflicts. As shown in Figure 3, airplanes *i* ∈ *I* and *i*′ ∈ *I* use the same gate consecutively, and the usage time periods of the two airplanes [*a*_*i*_, *d*_*i*_] and [*a*_*i*′_, *d*_*i*′_] should not overlap. Besides, buffer time *τ*_*b*_ should also be satisfied between serving two airplanes for ground operations. Secondly, because gates in terminal and satellite halls may have different functions (such as check-in facilities and passport control), we consider the gate compatibility in this study. In particular, for airplanes, we consider gate compatibility for wide/narrow-body types; for related flights, the gate compatibility is associated with serving domestic/international flights.

The gate assignment problem (GAP) is to assign airplanes *i* ∈ *I* to gates or apron *g* ∈ *G*∪*G*′ with considering constraints such as gate time conflict constraints and gate compatibility, and the objective function mainly concerns making efficient use of gates or reducing the number of occupied gates. The decision variables are binary gate assignment variables *x*_*ig*_,   *i* ∈ *I*,  *g* ∈ *G*, and binary gate utilization variables *x*_*g*_,   *g* ∈ *G*. In particular, *x*_*ig*_ equals 1 if airplane *i* is assigned to gate *g* and otherwise equals 0; *x*_*g*_ equals 1 if gate *g* is used by any airplane and otherwise equals 0.

The article "Managing the Gate Assignment Problem in the Hub Airport with Satellite Halls: A Transfer Demand-Oriented Approach" was retracted in 2023. Reasons: unreliable results or conclusions; concerns about the data; concerns about the peer review; concerns about the citations.

We also attempt to consider the impact of gate assignment on passengers in this study. The set of passenger groups is denoted by *P*. As shown in Figure 4, each group of passengers *p* ∈ *P* transfers from the same arrival flight served by airplane *i*_*p*_^1^ ∈ *I* to the same departure flight served by airplane *i*_*p*_^2^ ∈ *I* (which can be abbreviated as *i*_1_ and *i*_2_). The transfer time budget for passenger group *p* is defined as *B*_*p*_=*d*_*i*_2__ − *a*_*i*_1__. The number of passengers in group *p* is given and denoted by *n*_*p*_.

Gate assignment determines passengers' shortest transfer time, including processing time, walking time, and MRT time. It will affect passengers' transfer in the airport, especially hub airports with satellite halls. The layout in Figure 1 is taken as an example, and a passenger whose transfer time budget is 60 min is considered. Different transfer scenarios are illustrated in Table 2 when arriving and departing airplanes are assigned to different gates. In Scenario 1, both gates of arriving and departing airplanes are assigned in terminal *T*, and the shortest transfer time is much less than the transfer time budget *B*_*p*_ and transfer success. Passenger transfer is more stressful in Scenario 2 because the assigned gates of two airplanes are located at *T* and S1, respectively. Passengers in Scenario 3 and Scenario 4 fail to transfer due to the gate assignment.

Thus, passengers *p* may fail to transfer if the shortest transfer time is too long between two gates assigned to airplanes *i*_1_ and *i*_2_, i.e., exceeding the transfer time budget *B*_*p*_. The demand-oriented gate assignment problem (TGAP) in this study focuses on the trade-off between transfer passenger service and gate utilization efficiency in GAP when satellite halls are constructed in the hub airport.

### 2.2. Assumptions

To facilitate the presentation of our studied problem in this study, the following assumptions are made:

 
**A1**: (airport layout). Considering a hub airport with one terminal, several satellite halls, and an apron, the shortest transfer time between any two gates is given. There is no limit on the number and type of airplanes that use the apron simultaneously.
 
**A2**: (flight and airplane). Given the flight timetable in the research period, including arrival/departure time, flight types (domestic/international), and airplane types (wide/narrow-body).
 
**A3**: (gate service). Only one airplane can use a gate at a time. All of the gates have the same buffer time *τ*_*b*_ between serving two airplanes. The gate compatibility for flights and airplanes is considered.
 
**A4**: (passenger demand). Since the satellite halls mainly affect transfer passengers, it is assumed that we only consider the transfer passenger demand. The quantity, associated flights, and transfer time budget of passengers are given.

The article "Managing the Gate Assignment Problem in the Hub Airport with Satellite Halls: A Transfer Demand-Oriented Approach" was retracted in 2023. Reasons: unreliable results or conclusions; concerns about the data; concerns about the peer review; concerns about the citations.

## 3. Mathematical Formulation

In this section, we first formulate the model for GAP to clarify the resource utilization and constraints in the hub airport, and then, we propose the model for TGAP considering the service of transfer passengers in Section 3.2.

### 3.1. Notations and Decision Variables

Table 3 lists general indices, sets, parameters, and variables in optimization models that appeared in this study.

### 3.2. Model for GAP

In this subsection, the mathematic model of GAP is formulated to integrate using the gates in terminal and satellite halls, including constraints and multi-objective functions.

#### 3.2.1. Constraints

The constraints of GAP usually include gate utilization and airplane service, which are next described in detail.

*(1) Gate Time Conflict Constraint*. A feasible gate assignment scheme should guarantee that airplanes assigned to the same gate do not overlap in time and observe the buffer time. The airplane time incidence parameter *δ*_*it*_ is introduced, which equals 1 when *a*_*i*_ ≤ *t* ≤ *d*_*i*_+*τ*_*b*_ and otherwise 0. So, we have the following:

(1) $$\begin{array}{c} \underset{i\in I}{\sum }\delta_{it}\cdot x_{ig}\leq 1,\;\forall t\in T,\;\forall g\in G. \end{array}$$

The incidence parameter *δ*_*it*_ and assignment variable *x*_*ig*_ associate airplanes, gates, and time.

*(2) Gate Utilization Constraints*. For gate *g* ∈ *G*, if it is used by any airplane, the variable *x*_*g*_ equals 1, otherwise 0. So, we have gate utilization constraints that indicate the relationship between *x*_*ig*_ and *x*_*g*_ as follows:

(2) $$\begin{array}{c} \underset{i\in I}{\sum }x_{ig}\leq M\cdot x_{g},\;\forall g\in G, \end{array}$$

where *M* is a sufficiently large positive constant.

*(3) Airplane Service Constraints.* Each airplane must and can only be assigned to one gate or the apron, and then:

(3) $$\begin{array}{c} \sum_{g\in G\cup^{}G^{\prime }}x_{ig}=1,\;\forall i\in I. \end{array}$$

*(4) Gate Compatibility Constraints*. We consider the gate compatibility in this model, because gates in the different areas of terminal and satellite halls may have different functions, which are mainly influenced by facilities and equipment. The airplane gate compatibility incidence parameter *σ*_*ig*_ is introduced, which equals 1 if airplane *i* ∈ *I* can be served by gate *g* ∈ *G* and otherwise 0. We can derive the values of *σ*_*ig*_ based on the given airplane and gate types.

(4) $$\begin{array}{c} x_{ig}\leq \sigma_{ig},\;\forall i\in I,\;\forall g\in G\cup^{}G^{\prime }. \end{array}$$

In particular, the apron can serve all types of airplanes and *σ*_*ig*_=1,  *g* ∈ *G*′.

*(5) Constraints for Decision Variables.*

(5) $$\begin{array}{c} x_{ig}=\left\{\begin{array}{cc} 1\; & \text{if airplane i is assigned to gate }g\text{,}\\ 0 & \text{otherwise,} \end{array}\right.\;\forall i\in I,\forall g\in G\cup^{}G^{\prime },\\ x_{g}=\left\{\begin{array}{cc} 1 & \text{if gate }g\text{ is used,}\\ 0 & \text{otherwise,} \end{array}\right.\;\forall g\in G. \end{array}$$

Constraints (5) and (6) are binary requirements on the decision variables.

The article "Managing the Gate Assignment Problem in the Hub Airport with Satellite Halls: A Transfer Demand-Oriented Approach" was retracted in 2023. Reasons: unreliable results or conclusions; concerns about the data; concerns about the peer review; concerns about the citations.

#### 3.2.2. Objective Function

Gates are the scarce resource in an airport, and operational efficiency depends on the utilization of this bottleneck resource. Since the hub airport has terminal and satellite halls simultaneously, the GAP aims to make efficient use of the gates in the terminal and satellite halls and minimizes the operating costs.

An airplane can use parking positions in the apron if it cannot be assigned to a gate, but the apron is usually far away from the terminal and satellite halls, and passengers need to take a shuttle bus between the terminal and the apron. This will increase the transfer time of passengers on the one hand and increase the operating costs of the airport on the other hand. To make efficient use of the gates and avoid assigning airplanes to the apron, the first objective is to minimize the number of airplanes assigned to the apron:

(6) $$\begin{array}{c} \min Z_{1}=\sum_{i\in I}\sum_{g\in G^{\prime }}x_{ig}. \end{array}$$

This is a common objective in the literature of GAP (Ding et al. [6], Dorndorf et al. [7, 8], Drexl and Nikulin [9], Deng et al. [10]). It is equivalent to maximizing the number of airplanes assigned to gates. Furthermore, this objective can be easily extended to maximize the total usage time of gates since the dwell time of each airplane is given, but it has no significant impact on passenger service so we use the objective (6) in this study.

Besides, the GAP is multi-objective in nature and operation costs for gates are expensive (including ground operation costs), which motivates us to consider objectives more comprehensively. Apart from minimizing the apron operation, the GAP also needs to consider the objective that minimizes the number of used gates, i.e.,

(7) $$\begin{array}{c} \text{min}Z_{2}=\sum_{g\in G}x_{g}. \end{array}$$

In this study, we consider the objective function that consists of the number of airplanes assigned to the apron and the number of used gates and then formulate the GAP as a multi-objective optimization problem. For GAP in a hub airport with the apron, if we only consider the objective (6), gate operating hours may not be fully utilized in some situations; only consider the objective (7) is obviously not feasible either, which would assign all of the airplanes to the apron. Thus, the combination and trade-off between objectives (6) and (7) is comprehensive for GAP. We use linear weight to handle these two objectives and formulate the objective function as follows:

(8) $$\begin{array}{c} \text{min}Z_{\text{GAP}}=\alpha_{1}\cdot Z_{1}+\alpha_{2}\cdot Z_{2}, \end{array}$$

where *α*_1_ and *α*_2_ are positive weights to denote the trade-off between objectives. In particular, we can obtain a Pareto-optimal solution if *α*_1_ and *α*_2_ are set 1, or their values are set according to the preference of airport operators.

The article "Managing the Gate Assignment Problem in the Hub Airport with Satellite Halls: A Transfer Demand-Oriented Approach" was retracted in 2023. Reasons: unreliable results or conclusions; concerns about the data; concerns about the peer review; concerns about the citations.

#### 3.2.3. Mathematical Model for GAP

The GAP can be formulated as follows:

(9) $$\begin{array}{c} \left\{\begin{array}{c} \text{min}Z_{\text{GAP}}=\alpha_{1}\cdot \sum_{i\in I}\sum_{g\in G^{\prime }}x_{ig}+\alpha_{2}\cdot \sum_{g\in G}x_{g},\\ s.t.\;\text{constraints}\;\left(1\right)-\left(6\right). \end{array}\right. \end{array}$$

The mathematical model for GAP given in (9) is binary integer linear programming. The model for GAP focuses on the gate resource optimization when a hub airport has both main terminal and satellite halls, and next, we will consider the impact of GAP on passengers and further improve the model involving different stakeholders.

### 3.3. Model for TGAP

Gate assignment affects the service quality of passengers, especially the transfer passengers in the hub airport where both main terminal and satellite halls are providing passenger service. Passengers may take a longer time to get from the arriving flight to the departing flight gate due to the gate assignment and may even exceed the transfer time budget resulting in a failed transfer. Thus, we will incorporate the service of transfer passengers in the GAP in this section.

With the given flight timetable and transfer scheme (arriving airplane *i*_1_ and departing airplane *i*_2_) of passenger group *p* ∈ *P*, we can get the transfer time budget *B*_*p*_=*d*_*i*_2__ − *a*_*i*_1__. The gates serving airplanes *i*_1_ and *i*_2_ are denoted as *g*_1_ and *g*_2_, respectively. Given the layout of terminal and satellite halls in the airport, the shortest transfer time *τ*(*g*_1_, *g*_2_) (including processing time, walking time, and MRT time) between any two gates is also fixed.

The article "Managing the Gate Assignment Problem in the Hub Airport with Satellite Halls: A Transfer Demand-Oriented Approach" was retracted in 2023. Reasons: unreliable results or conclusions; concerns about the data; concerns about the peer review; concerns about the citations.

The gate assignment will influence the shortest transfer time of passenger group *p*. Here, we introduce the transfer pressure to describe the airport's service level for transfer passengers. The transfer pressure is the ratio of shortest transfer time to transfer time budget, and the transfer pressure for passenger *p* is denoted by *φ*_*p*_ and defined as follows:

(10) $$\begin{array}{c} \varphi_{p}=\left\{\begin{array}{cc} \frac{\tau \left(g_{1},g_{2}\right)}{B_{p}}, & \text{ if }i_{1},i_{2}\text{ are both assigned to gates},\\ \frac{\tau_{c}}{B_{p}}, & \text{ otherwise}, \end{array}\right. \end{array}$$

where *τ*_*c*_ is the total transfer time (including process time and shuttle bus time) for passengers associated with the apron. If both associate airplanes of a passenger group are assigned to gates in the terminal and satellite halls, passengers need to do a gate-gate transfer with transfer time *τ*(*g*_1_, *g*_2_); otherwise, passengers need to do a gate-apron, apron-gate, or even apron-apron transfer with transfer time *τ*_*c*_. Note that *τ*_*c*_ is longer than the shortest transfer time between any two gates because the parking positions in the apron are usually far away from the terminal and satellite halls.

Then, we introduce the objective that minimizes the transfer pressure for passengers to capture the passenger service in the GAP of the hub airport; i.e.,

(11) $$\begin{array}{c} \text{min}Z_{3}=\sum_{p\in P}\sum_{g_{1}\in G\cup^{}G^{\prime }}\sum_{g_{2}\in G\cup^{}G^{\prime }}x_{i_{1}g_{1}}x_{i_{2}g_{2}}\varphi_{p}n_{p}. \end{array}$$

The GAP considering passenger transfer time budget can be formulated as follows:

(12) $$\begin{array}{c} \left\{\begin{array}{c} \text{min}Z_{\text{TGAP}}=\alpha_{1}\cdot \sum_{i\in I}\sum_{g\in G^{\prime }}x_{ig}+\alpha_{2}\cdot \sum_{g\in G}x_{g}+\alpha_{3}\cdot \sum_{p\in P}\sum_{g_{1}\in G\cup^{}G^{\prime }}\sum_{g_{2}\in G\cup^{}G^{\prime }}x_{i_{1}g_{1}}x_{i_{2}g_{2}}\varphi_{p}n_{p},\\ s.t.\;\text{constraints}\;\left(1\right)-\left(6\right). \end{array}\right.. \end{array}$$

The mathematical model given in (12) explicitly considers the transfer passenger service and shows the trade-off between passenger service and operating costs of GAP in the hub airport. The mathematical model (12) is nonlinear programming, and the nonlinearities come from the objective function associated with passenger, where the calculation of transfer pressure *φ*_*p*_ is a segmentation function.

Table 4 presents the complexity of the model for GAP and TGAP. It can be seen that the model size depends on the number of gates, airplanes, passenger groups, and demand discretization (number of discretized time intervals). Suppose that there is a hub airport with 10 gates and 100 airplanes with 100 transfer passenger groups, the research period is [0 : 00 − 24 : 00]. If the discretization time interval is 5 min, there will be 120 variables and 2500 constraints in the GAP model (9). The number of variables in the TGAP model (11) is 1120, with the addition of variables related to transfer passengers.

The article "Managing the Gate Assignment Problem in the Hub Airport with Satellite Halls: A Transfer Demand-Oriented Approach" was retracted in 2023. Reasons: unreliable results or conclusions; concerns about the data; concerns about the peer review; concerns about the citations.

## 4. Solution Approach

The mathematic model (9) for GAP is a binary integer linear programming and can be solved by several existing commercial solvers, such as CPLEX and Gurobi (see, e.g., Linderoth and Ralphs [27]; Atamturk and Savelsbergh [28]).

As for the mathematic model (12) for TGAP, it is nonlinear programming with linear constraints, and we next propose two approaches to solve it.

### 4.1. Linearization Approach

In this section, the origin nonlinear programming model (12) will be transformed into binary integer linear programming by introducing new binary variables and linear constraints.

Focusing on the nonlinear objective function of the model (12), the calculation of transfer pressure *φ*_*p*_ is a segmentation function as shown in Eq. (11). According to the analysis of transfer time under different scenarios in Section 3.3, only need to set the shortest transfer time associated with *g* ∈ *G*′ as *τ*_*c*_, i.e., *τ*(*g*_1_, *g*_2_)=*τ*_*c*_, *g*_1_ ∈ *G*′ or *g*_2_ ∈ *G*′ the objective that minimizes the transfer pressure in (12) could be updated as follows:

(13) $$\begin{array}{c} \text{min}Z_{3}=\sum_{p\in P}\sum_{g_{1}\in G\cup^{}G^{\prime }}\sum_{g_{2}\in G\cup^{}G^{\prime }}\frac{x_{i_{1}g_{1}}x_{i_{2}g_{2}}\tau \left(g_{1},g_{2}\right)n_{p}}{B_{p}}. \end{array}$$

It can be observed that (13) is nonlinear because of productions of binary variables *x*_*i*_1_*g*_1__ and *x*_*i*_2_*g*_2__, and they can be replaced by auxiliary binary variables *y*_*i*_1,2_*g*_1,2__. Following Williams [29], the productions can be replaced by adding linear constraints:

(14) $$\begin{array}{c} \left\{\begin{array}{c} -x_{i_{1}g_{1}}+y_{i_{1,2}g_{1,2}}\leq 0\\ -x_{i_{2}g_{2}}+y_{i_{1,2}g_{1,2}}\leq 0\\ x_{i_{1}g_{1}}+x_{i_{2}g_{2}}-y_{i_{1,2}g_{1,2}}\leq 1\\ y_{i_{1,2}g_{1,2}}\in \left\{0,1\right\} \end{array}\right.,\;\forall p\in P,\;\forall g_{1},g_{2}\in G. \end{array}$$

Thus, the linearized model for TGAP considering the transfer passenger service can be formulated as follows:

(15) $$\begin{array}{c} \left\{\begin{array}{c} \text{min}Z_{\text{TGAP}}=\alpha_{1}\cdot \sum_{i\in I}\sum_{g\in G^{\prime }}x_{ig}+\alpha_{2}\cdot \sum_{g\in G}x_{g}+\alpha_{3}\cdot \sum_{p\in P}\sum_{g_{1}\in G\cup^{}G^{\prime }}\sum_{g_{2}\in G\cup^{}G^{\prime }}\frac{y_{i_{1,2}g_{1,2}}\tau \left(g_{1},g_{2}\right)n_{p}}{B_{p}},\\ s.t.\;\text{constraints}\left(1\right)-\left(6\right),\left(14\right). \end{array}\right.. \end{array}$$

Note that model (15) is linear programming and can easily be solved by commercial solvers such as CPLEX and Gurobi to find a globally optimal solution.

The article "Managing the Gate Assignment Problem in the Hub Airport with Satellite Halls: A Transfer Demand-Oriented Approach" was retracted in 2023. Reasons: unreliable results or conclusions; concerns about the data; concerns about the peer review; concerns about the citations.

As shown in Table 4, the number of auxiliary binary variables *y*_*i*_1,2_*g*_1,2__ is |*P*| × (|*G*|+1)^2^. Based on the example in Section 3, there will be 121120 variables and 489000 constraints in the linearized model (15) for TGAP. Besides, when the number of passenger groups and airport gates increases, the number of variables and constraints increases rapidly, which takes a long computation time to solve the TGAP with commercial solvers. To address this issue, we further design a heuristic approach to solve the TGAP.

### 4.2. Heuristic Approach

The gate assignment problem is a complex nondeterministic polynomial hard (NP-hard) problem due to the complex layout of airports, multi-flights, passenger trips, and gate compatibility [30, 31], and many studies adopted heuristic approaches to solve it [16, 21, 24]. To solve TGAP in large hub airports requires an efficient algorithm to obtain a satisfactory solution and solve the problem in reasonable CPU time. The simulated annealing (SA) algorithm is a metaheuristic to approximate the global optimization and has good robustness. Thus, we propose an approach for TGAP at large hub airports based on the framework of the SA algorithm.

In Algorithm 1, we adopt the following strategies to adjust the assignment scheme and get neighborhood solutions.

#### 4.2.1. Initial Solution

The model (11) for TGAP has the same constraints as the model (9) for GAP, and we can use the optimal solution of model (9) as the initial solution. It is already efficient in terms of gate resource utilization. As for the model scales, note that the model (9) can be decomposed into two subproblems by gate compatibility on airplane types: one assignment for wide-body airplanes and associate gates and another for narrow-body airplanes and associate gates. In this way, the initial solution of TGAP is designed.

#### 4.2.2. Passenger Service Adjustment Strategy

The passenger service adjustment strategy aims to reduce the transfer pressure of passengers, which includes three options: insert option, swap operation, and remove operation. These operations are performed sequentially, with only one of them executed in each loop, and detailed options are shown as follows.

The article "Managing the Gate Assignment Problem in the Hub Airport with Satellite Halls: A Transfer Demand-Oriented Approach" was retracted in 2023. Reasons: unreliable results or conclusions; concerns about the data; concerns about the peer review; concerns about the citations.

In the current solution, we already know the gate assignment scheme, i.e., the specific gate of each airplane. As we know the transfer information of passenger group *p* ∈ *P*, *P*_*i*_^1^ and *P*_*i*_^2^ are denoted as the subset of passenger groups whose arriving and departing airplane is *i* ∈ *I*, respectively. Then, we denote *φ*_*i*_ as the total transfer pressure of passengers associated with airplane *i*, which is given as follows:

(16) $$\begin{array}{c} \varphi_{i}=\sum_{p\in P_{i}^{1}}\varphi_{p}n_{p}+\sum_{p\in P_{i}^{2}}\varphi_{p}n_{p}. \end{array}$$

The total transfer pressure of each airplane is calculated by equation (16) and does the following operations: ① the airplane that has the maximum transfer pressure and is already assigned to a gate is selected. ② Insert operation: the subset of gates that has available time and already been used is found, the selected airplane is inserted into one of them randomly. If the subset is empty, the next operation is proceeded. ③ Swap operation: the subset of airplanes that has the same time interval and type (no violation of constraints (1) and (4)) is found, the selected airplane and one of them are randomly swapped. If the subset is empty, the next operation is proceeded. ④ Remove operation: if the above two operations are not executed, the subset of gates suitable for the selected airplane is found, one of them is chosen at random, and the selected airplane is assigned to this gate, and then, the airplanes with conflicts are assigned to the apron.

#### 4.2.3. Gate Utilization Strategy

The gate utilization strategy concentrates on reducing the number of used gates, which includes two options: insert option and remove operation. Based on the current solution, we could know the set of airplanes assigned to gate *g* ∈ *G* and denoted by *I*_*g*_. *u*_*g*_ is denoted as the time utilization ratio of gate *g*, which equals the ratio of occupied time to research period:

(17) $$\begin{array}{c} u_{g}=\sum_{i\in I_{g}}\frac{\left(\tau_{b}+d_{i}-a_{i}\right)}{\left(T_{2}-T_{1}\right)}. \end{array}$$

To reduce the number of used gates, the following operations are executed: ①the gate with the lowest time utilization ratio using (17)is found, and if the ratio is lower than a threshold value (such as 40%), then next options are done. ② insert operation: for airplanes assigned to the selected gate, the subset of gates that has available time and already used is found, and these airplanes are inserted in one of them randomly. ③ Remove operation: the rest of the airplanes are assigned to the apron after the previous option.

#### 4.2.4. Apron Airplane Adjustment Strategy

The apron airplane adjustment strategy is designed to reduce the number of airplanes assigned to the apron and transfer pressure of passengers. Thus, included operations in this part of the strategy consider both of the two objectives. ① The total transfer pressure of each airplane in the apron by (16)is calculated and the maximum one of them is found. ② The insert and swap operations are executed. This airplane is randomly inserted into a gate that has available time periods; otherwise, it is swapped with another airplane assigned to a gate without violation of constraints (1) and (4). ③ If the above two operations are not satisfied, one of the airplanes in the apron is attempted insert into an available gate. ④ If there is any available empty gate, the airplane with the shortest overlap time period with other airplanes in the apron is found and assigned to the new gate.

The article "Managing the Gate Assignment Problem in the Hub Airport with Satellite Halls: A Transfer Demand-Oriented Approach" was retracted in 2023. Reasons: unreliable results or conclusions; concerns about the data; concerns about the peer review; concerns about the citations.

The proposed heuristic approach shown in Algorithm 1 is based on the framework of the SA algorithm, together with three strategies for improving different parts of objective functions, and it would find a satisfactory solution of TGAP in the model (13).

## 5. Case Studies

To demonstrate the performance of the proposed models and solve approaches, we use the data of the Shanghai Pudong International Airport in China as a case study. We will describe the experiment data in Section 5.1. The numerical results are presented in Section 5.2.

All numerical tests are conducted on a personal computer with Intel® Core (™) 3.00 GHz processor and 16.00 GB RAM and Windows 10 Home Edition Operating System (64 bit). The YALMIP-R20190425 together with MATLAB R2019b is used to conduct the numerical tests. The commercial solver Gurobi optimization studio 8.1.1 (with academic license) is adopted to solve GAP and linearized TGAP models, and the solver used the branch-and-cut algorithm to find optimal solutions for the above two mixed-integer programming models.

### 5.1. Data and Parameter Setting

We consider a real-world case study on the Shanghai Pudong International Airport, which is an important hub airport in eastern China. The gates are integrated used in a terminal *T* and connected satellite hall S, and both terminal *T* and satellite hall S could handle transfer processes for passengers. There is an MRT line that connects *T* and S to quickly transport passengers, assuming that passengers' MRT time for a one-way trip is 5 minutes (for layout, see Figure 5). We consider the GAP and TGAP for 28 gates in terminal *T* and 41 gates in satellite hall S and an apron, and the detailed information of gates can be found in Table 5. The compatibility of gates such as service for domestic/international flights and wide/narrow-body airplanes is also given. *τ*_*c*_ is set as 180 minutes.

The article "Managing the Gate Assignment Problem in the Hub Airport with Satellite Halls: A Transfer Demand-Oriented Approach" was retracted in 2023. Reasons: unreliable results or conclusions; concerns about the data; concerns about the peer review; concerns about the citations.

In this case study, the considered research period is set as [0 : 00 − 24 : 00], which covers a full day of operations. We select 296 airplanes related to the above gates of China Eastern Airlines and Xiamen Airlines on January 20, 2018.  Table 6 shows several records as an example, and every record corresponds to one airplane, which services two flights. The information of airplanes includes the arrival and departure date, arrival and departure time, arrival and departure flights, airplane types (wide/narrow-body), and flight types (domestic/international).

Meanwhile, transfer information of more than 3000 passengers is selected and divided into groups based on arrival and departure flights. The example of information is shown in Table 7, which includes arrival and departure flight, arrival and departure date, and passenger number in groups. Combining with the information of airplanes and flights in Table 6, we can easily get the transfer time budget of each passenger group. Since the layout of the airport is set, the shortest transfer time *τ*(*g*_1_, *g*_2_) between any two gates is also determined, including processing time, walking time, and MRT time. The buffer time of gates *τ*_*b*_ is set to 45 minutes.

The linear weights in the model (10), (13), and (16) are, respectively, *α*_1_=296,  *α*_2_=1,  *α*_3_=10; the algorithm parameters are set as follows: *T*_0_=10^6^,   *T*_*f*_=5, *m*_max_=50, *θ*=0.5.

### 5.2. Computational Results

Given the above data and settings, the proposed solution approaches will be implemented for GAP and TGAP. The results of GAP, TGAP with linearization approach, and performance comparison are shown in Subsection 5.2.1; Subsection 5.2.2 shows the result of TGAP solved by the heuristic approach.

#### 5.2.1. Solutions of GAP and Linearized TGAP

In this subsection, we solve the GAP and linearized TGAP by commercial solver Gurobi optimization, and the CPU time to solve GAP is 5.75s. The result of GAP is shown in Figure 6, and the horizontal axis represents the research period ([0 : 00 − 24 : 00] on January 20, 2018), and the vertical axis represents the total of 69 gates in terminal *T* and satellite hall S. The colored bars in Figure 6 represent the time period when the airplanes occupy the corresponding gates, and the buff time is not included. It can be clearly seen that airplanes satisfy the time conflict constraints of gates and buffer time is also held between two adjacent airplanes. One can find that airplanes arriving and departing during [0 : 00 − 6 : 00] usually occupy the gates for a long time as passengers tend not to travel at this period. The result of TGAP is shown in Figure 7, which also satisfies all of the constraints.

The article "Managing the Gate Assignment Problem in the Hub Airport with Satellite Halls: A Transfer Demand-Oriented Approach" was retracted in 2023. Reasons: unreliable results or conclusions; concerns about the data; concerns about the peer review; concerns about the citations.

From Figure 6, we can find that several gates (S29, S30, S39, and S41) are not occupied by any airplane, and they are all serving wide-body airplanes. Meanwhile, Figure 8 shows that all wide-body airplanes are already assigned to gates in GAP and that ratio for narrow-body airplanes is 81%, and the total number of airplanes successfully assigned to the gates is 249. Here is why we consider the objective that minimizes the number of used gates in (7), which can improve the efficiency of gate utilization when one kind of resource is sufficient, i.e., gates for wide-body airplanes. Thus, the combination of objectives (6) and (7) is more comprehensive for gate utilization in both GAP and TGAP.

Next, we compare the solution of GAP and TGAP, and values of different parts in objective functions are shown in Table 8, of which the value of *Z*_3_ (transfer pressure) in GAP is calculated based on the optimal solution of the model (10) and services for passengers are not taken into account. It is obvious from Table 8 that when the first and second objectives (minimizing the number of apron airplanes *Z*_1_ and used gates *Z*_2_) are close in the GAP and TGAP, considering the objective *Z*_3_ can significantly reduce the transfer pressure of passengers (23.64% reduction). That is, model (12) of the TGAP can improve the service level of transfer passengers without increasing the resource requirement in the hub airport. Moreover, although the number of assigned airplanes has decreased in the TGAP solution, the time utilization rate of gates in terminal *T* and satellite hall S has increased, and the scheme in TGAP assigns airplanes serving more transfer passengers and with less occupation time to the gates. This also demonstrates that considering the gate resource utilization and passenger service simultaneously is a more comprehensive way to address gate assignment in the hub airport.

#### 5.2.2. Solution of TGAP Adopting Heuristic Approach

Although the proposed linearization approach in Section 4.1 can obtain the global optimal solution for TGAP, it takes a long time to converge. We adopted the commercial solver Gurobi optimization studio 8.1.1 to solve the linearized TGAP, and the CPU time to get the optimal solution is 6.09 h. The proposed heuristic approach takes 726s to solve the TGAP with the same input and parameters and only has a 2.59% solution GAP with linearization approach, and the gate assignment scheme is shown in Figure 9 as follows.

Passenger group no. 3 in Table 7 is taken as an example, passenger transfers from flight MU5698 arriving on January 20, 14:30, to flight MU545 departing at January 20, 16:10, and the transfer time budget is 100 min. In the GAP solution, airplanes separately serving the arrival and departure flight are assigned to gates S5 and T3. As the two gates are not in the same terminal, the shortest transfer time for passengers is 60 min. When we take the transfer pressure into account in TGAP, the above two airplanes are assigned to gates T18 and T5, which are both in the terminal *T*, passengers' shortest transfer time reduced to 35 min, and transfer pressure decreased from 0.60 to 0.35. Furthermore, the total transfer pressure of passengers in the solution of TGAP by the heuristic approach is still lower than that in the solution of GAP. This indicates that the TGAP well considered the service for passengers and realized the integrated assignment of gates in terminal and satellite halls.

The article "Managing the Gate Assignment Problem in the Hub Airport with Satellite Halls: A Transfer Demand-Oriented Approach" was retracted in 2023. Reasons: unreliable results or conclusions; concerns about the data; concerns about the peer review; concerns about the citations.

As shown in Figure 10, gates in the terminal *T* are all used due to the shorter transfer time related to the gates in *T* than that in S, and there are 3 gates in the satellite hall S serving wide-body airplanes that are not used. The total utilization rate of gates is 96%, and the time utilization rate is 69.98%. For TGAP, although the gate time utilization rate in the solution of the linearized approach (70.21%) is higher than that of the heuristic approach, the difference is not significant.

Next, we compare the passenger transfer pressure in three cases: the GAP solution, linearized approach of TGAP solution, and heuristic approach of TGAP solution. The proportion of passengers within different transfer pressure intervals of the above three solutions are reported in Figure 11, where we observe that most of the passengers' transfer pressure remains at a relatively low level and lies in the range of [0.1, 0.5] in all three cases. Two solutions of TGAP are compared with the GAP solution, and we can see that the quantity of passengers who experience low transfer pressure ([0.1, 0.3]) in TGAP solutions is significantly more than that in the GAP solution, while in the high transfer pressure range ([0.5, 1.0]), the proportion of passengers in TGAP solutions is less than that in the GAP solution. This result indicates that proposed TGAP models could improve the service for transfer passengers.

Turning now to solutions of TGAP by linearization approach and heuristic approach, the distributions of passenger transfer pressure in these two solutions are comparable, which means the proposed heuristic approach could obtain a satisfactory solution in a reasonable time. What is striking in Figure 11 is that some passengers in all three solutions have transfer pressure greater than 1 because related airplanes are assigned to the apron, and this situation is enhanced in TGAP solutions.

The article "Managing the Gate Assignment Problem in the Hub Airport with Satellite Halls: A Transfer Demand-Oriented Approach" was retracted in 2023. Reasons: unreliable results or conclusions; concerns about the data; concerns about the peer review; concerns about the citations.

## 6. Conclusions and Future Research

In this study, we focus on the impacts of gate assignment on the service of transfer passengers in the hub airport with satellite halls. First, a binary linear programming model for GAP is proposed that considers the gate time conflict, gate compatibility constraints, and the airport operator-oriented objective functions. Then, we introduce the transfer time budget and transfer pressure to measure the passenger service and formulate the TGAP as a nonlinear programming with linear constraints. In particular, multi-objective functions were considered in the TGAP model, including transfer demand-oriented and operator-oriented objectives. We proposed a linearization approach and a SA algorithm-based heuristic approach to solve the nonlinear model of TGAP. Finally, the case study based on practical data demonstrated the benefits of the proposed models and solution approaches. In the experimental results, it was verified that the proposed TGAP model and solution approaches can improve the service for transfer passengers and lead to more efficient utilization of gate resources in the hub airport.

Further research could consider the randomness of transfer passenger demand and the effects of random flight delay on gate assignment and transfer passenger service. We can also manage the fairness of passengers through transfer pressure in the gate assignment problem.

## Figures and Tables

**Figure 1:** Example layout of the hub airport with satellite halls.

**Figure 2:** Airplane and served flights.

**Figure 3:** Gate utilization and buffer time.

**Figure 4:** Illustration for transfer time budget of passengers.

**Figure 5:** Layout of terminal T1 and satellite hall S1 in Shanghai Pudong International Airport.

**Figure 6:** Optimal gate assignment scheme of GAP.

**Figure 7:** Optimal gate assignment scheme of linearized TGAP.

**Figure 8:** Assigned numbers and rates for different types of airplanes in GAP.

**Figure 9:** Gate assignment scheme of TGAP solved by the heuristic approach.

**Figure 10:** Gate utilization in terminal T and satellite hall S in TGAP.

**Figure 11:** Comparison of passenger transfer pressure.

**Algorithm 1:** Solving framework based on SA algorithm for TGAP.

**Table 1:** Comparisons of major-related studies.

Paper	Airport-orainted objective	Passenger-orainted objective	Transfer passenger	Gate compatibility	Solution method
Bihr [19]	—	Walking distance	No	—	Simplex algorithm
Ding et al. [6]	Unassigned airplane	Walking distance	Yes	—	Tabu search
Yan and Tang [24]	—	Waiting time	No	—	Heuristic approach
Drexl and Nikulin [9]	Unassigned airplane and flight-gate preferences	Walking distance	Yes	—	Pareto SA
Dell'orco et al. [21]	Unassigned airplane	Walking distance	Yes	—	Bee Colony Algorithms
Das [26]	Passengers assigned to specific gates	Walking distance	No	—	Two phase local search
Deng et al. [30]	Gate utilization	Walking distance	Yes	Airplane type	Quantum evolutionary algorithm
This paper	Unassigned airplane and gate utilization	Transfer pressure	Yes	Airplane and flight type	Linearization approach and SA-based algorithm

The article "Managing the Gate Assignment Problem in the Hub Airport with Satellite Halls: A Transfer Demand-Oriented Approach" was retracted in 2023. Reasons: unreliable results or conclusions; concerns about the data; concerns about the peer review; concerns about the citations.

**Table 2:** Transfer scenarios for passenger group *p* under different gate assignment schemes.

Scenarios	Gate of arriving airplane	Gate of departing airplane	Shortest transfer time	Transfer time budget *B*_*p*_	Result
1	Gate 1 (T)	Gate 2 (T)	30 min	60 min	Success
2	Gate 1 (T)	Gate 3 (S1)	55 min		Success
3	Gate 1 (T)	Gate 5 (S2)	70 min		Fail
4	Gate 1 (T)	Gate 7 (apron)	>70 min		Fail

**Table 3:** Main sets, indices, parameters, and variables.

Symbol	Definition
*Sets and indices*	
*G*	Set of gates in the terminal and satellite halls
*G*′	Set of parking positions in the apron
*I*	Set of airplanes
*P*	Set of passenger groups
*T*	Set of discretized time intervals
*g*	Index of all gates and parking positions, *g* ∈ *G*∪*G*′
*i*	Index of airplanes, *i* ∈ *I*
*p*	Index of passenger groups, *p* ∈ *P*
*t*	Index of discretized time intervals, *t* ∈ *T*

*Parameters*	
[*T*_1_, *T*_2_]	Daily operation period
*τ*_*b*_	Buffer time of gates
*a*_*i*_	Arrival time of airplane *i*
*d*_*i*_	Departure time of airplane *i*
*δ*_*it*_	Airplane time incidence parameter
*σ*_*ig*_	Airplane gate compatibility incidence parameter
*i*_*p*_^1^	Arriving airplane of passenger group *p*, abbreviated as *i*_1_
*i*_*p*_^2^	Departing airplane of passenger group *p*, abbreviated as *i*_2_
*B*_*p*_	Transfer time budget of passenger group *p*
*n*_*p*_	Number of passengers in group *p*
*τ*(*g*_1_, *g*_2_)	Shortest transfer time between gate *g*_1_ ∈ *G*∪*G*′ and *g*_2_ ∈ *G*∪*G*′
*τ*_*c*_	Waiting time for passengers when fail to transfer
*M*	A sufficiently large constant
*ε*	A sufficiently small positive constant
_c_	Weights in the objective function

Variables	
*x*_*ig*_	Binary assignment variable: *x*_*ig*_=1 if airplane *i* ∈ *I* is assigned to gate *g* ∈ *G*∪*G*′, and *x*_*ig*_=0, otherwise
*x*_*g*_	Binary utilization variable: *x*_*g*_=1 if gate *g* ∈ *G* is used, and *x*_*g*_=0, otherwise
*φ*_*p*_	Transfer pressure of passenger group *p*
*y*_*i*_1,2_ *g*_1,2__	Binary variable: *y*_*i*_1,2_*g*_1,2__=1 for passenger *p*, if arriving airplane *i*_1_ is assigned to *g*_1_ and departing airplane *i*_2_ is assigned to *g*_2_, and *y*_*i*_1,2_*g*_1,2__=0, otherwise

**Table 4:** Numbers of variables and constraints in the models.

Variables and constraints	Quantity
*Variables*	
*x*_*ig*_	|*I*| × |*G*|+|*I*|
*x*_*g*_	|*G*|
*φ*_*p*_	|*P*|
*y*_*i*_1,2_ *g*_1,2__	|*P*| × (|*G*|+1)^2^

*Constraints*	
Gate time conflict constraint (1)	|*T*| × |*G*|
Gate utilization constraints (2)	|*G*|
Airplane service constraints (3)	|*I*|
Gate compatibility constraints (4)	|*I*| × |*G*|+|*I*|
Binary constraints (5)	|*I*| × |*G*|+|*I*|
Binary constraints (6)	|*G*|

Note: |  ·  | represents the cardinality of a set.

The article "Managing the Gate Assignment Problem in the Hub Airport with Satellite Halls: A Transfer Demand-Oriented Approach" was retracted in 2023. Reasons: unreliable results or conclusions; concerns about the data; concerns about the peer review; concerns about the citations.

**Table 5:** Gate information and compatibility in the case study.

Gate no.	Terminal	Arrival service	Departure service	Airplane type	Gate no.	Terminal	Arrival service	Departure service	Airplane type
T1	T	I	I	N	S1	S	D	D	N
T2	T	I	I	W	S2	S	D	D	N
T3	T	I	I	W	S3	S	D	D	N
T4	T	I	I	W	S4	S	D	D	N
T5	T	I	D, I	W	S5	S	D	D	N
T6	T	D, I	D, I	W	S6	S	D	D	N
T7	T	D, I	D, I	N	S7	S	D	D	N
T8	T	D, I	D	N	S8	S	D	D	N
T9	T	D, I	D	N	S9	S	D	D	N
T10	T	D	D	N	S10	S	D	D	N
T11	T	D	D	N	S11	S	I	I	N
T12	T	D	D	N	S12	S	I	I	N
T13	T	D	D	N	S13	S	I	I	N
T14	T	D	D	N	S14	S	D	D	N
T15	T	D	D	N	S15	S	D	D	N
T16	T	D	D	N	S16	S	D	D	N
T17	T	D	D	N	S17	S	D	D	N
T18	T	D	D	N	S18	S	D	D	N
T19	T	D	D	N	S19	S	D	D	N
T20	T	D	D, I	N	S20	S	D	D	N
T21	T	D	D, I	N	S21	S	D	D	N
T22	T	D, I	D, I	N	S22	S	D	D	N
T23	T	D, I	D, I	W	S23	S	D	D	N
T24	T	D, I	D, I	W	S24	S	D	D	N
T25	T	D, I	I	W	S25	S	D	D	N
T26	T	I	I	W	S26	S	D	D	N
T27	T	I	I	W	S27	S	D	D	N
T28	T	I	I	W	S28	S	D	D	N
S29	S	D	D	W	S36	S	I	I	W
S30	S	D	D	W	S37	S	I	I	W
S31	S	I	I	W	S38	S	I	I	W
S32	S	I	I	W	S39	S	I	I	W
S33	S	I	I	W	S40	S	I	I	W
S34	S	I	I	W	S41	S	I	I	W
S35	S	I	I	W					

*Note.* T: terminal, S: satellite hall, D: domestic flight service, I: international flight service, W: wide-body airplane service, N: narrow-body airplane service.

**Table 6:** Partial airplane and flight records.

Airplane no.	Arrival flight number	Arrival date and time	Arrival type	Departure flight number	Departure date and time	Departure type	Airplane type
1	MU6753	Jan 19, 19:50	D	MU6358	Jan 20, 08:15	D	N
2	MU6785	Jan 20, 11:00	D	MU398	Jan 20, 13:10	I	N
3	MU6155	Jan 20, 13:20	I	MU6494	Jan 20, 14:25	D	N
4	MU663	Jan 20, 16:30	I	MU6588	Jan 20, 20:05	I	W
5	FM9188	Jan 20, 17:20	D	FM865	Jan 20, 18:20	I	N
6	MU5588	Jan 20, 21:20	D	MU5515	Jan 21, 08:55	D	N

*Note.* D: domestic flight, I: international flight, W: wide-body airplane, N: narrow-body airplane.

**Table 7:** Partial transfer passengers' information.

Passenger group no.	Number of passengers	Arrival flight number	Arrival date and time	Departure flight number	Departure date and time
1	10	MU5668	Jan 19, 18:35	MU739	Jan 20, 00:20
2	44	MU212	Jan 20, 10:20	MU207	Jan 20, 12:05
3	9	MU5698	Jan 20, 14:30	MU545	Jan 20, 16:10
4	20	MU504	Jan 20, 18:25	MU6720	Jan 20, 20:55
5	7	MU5130	Jan 20, 21:40	MU5023	Jan 21, 00:15

The article "Managing the Gate Assignment Problem in the Hub Airport with Satellite Halls: A Transfer Demand-Oriented Approach" was retracted in 2023. Reasons: unreliable results or conclusions; concerns about the data; concerns about the peer review; concerns about the citations.

**Table 8:** Performance comparison of GAP and linearized TGAP solutions.

Problem	*Z*_1_	*Z*_2_	*Z*_3_	Gate time utilization rate
GAP	47	65	1361.15^*∗*^	66.40%
TGAP	48	65	1039.31	70.21%

^*∗*^Note: the total passenger transfer pressure *Z*_3_ of GAP is calculated after solving the optimal solution.

## Data Availability

The practical data used to support the case study and findings in this study are available from the corresponding author upon request.
